The article "Dental Images' Segmentation Using Threshold Connected Component Analysis" was published in 2021. Journal: Comput Intell Neurosci.

# Dental Images' Segmentation Using Threshold Connected Component Analysis

**DOI:** 10.1155/2021/2921508

**Published:** 2021-12-14

**Authors:** Vincent Majanga, Serestina Viriri

**Affiliations:** School of Mathematics, Statistics and Computer Science, University of KwaZulu-Natal, Durban 4000, South Africa

## Abstract

Recent advances in medical imaging analysis, especially the use of deep learning, are helping to identify, detect, classify, and quantify patterns in radiographs. At the center of these advances is the ability to explore hierarchical feature representations learned from data. Deep learning is invaluably becoming the most sought out technique, leading to enhanced performance in analysis of medical applications and systems. Deep learning techniques have achieved great performance results in dental image segmentation. Segmentation of dental radiographs is a crucial step that helps the dentist to diagnose dental caries. The performance of these deep networks is however restrained by various challenging features of dental carious lesions. Segmentation of dental images becomes difficult due to a vast variety in topologies, intricacies of medical structures, and poor image qualities caused by conditions such as low contrast, noise, irregular, and fuzzy edges borders, which result in unsuccessful segmentation. The dental segmentation method used is based on thresholding and connected component analysis. Images are preprocessed using the Gaussian blur filter to remove noise and corrupted pixels. Images are then enhanced using erosion and dilation morphology operations. Finally, segmentation is done through thresholding, and connected components are identified to extract the Region of Interest (ROI) of the teeth. The method was evaluated on an augmented dataset of 11,114 dental images. It was trained with 10 090 training set images and tested on 1024 testing set images. The proposed method gave results of 93% for both precision and recall values, respectively.

## 1. Introduction

Dental caries is the most widespread chronic disease affecting teeth worldwide. Recently, there has been a decline in the rates of large cavity lesions, but still early lesions can be identified in most people [1]. Most of conventional caries detection methods rely on inspecting teeth visually. These methods are effective for large, clearly visible carious lesions as well as those partially visible but can be viewed by a handheld mirror [2]. The introduction of dental radiography is to detect hidden or inaccessible lesions that could not be otherwise done through conventional methods. Early detection of dental caries lesions is an important determinant of treatment measures and is therefore a beneficiary of the introduction of new tools [3]. The fastest growing sectors in the health care industry are dental services which consist of prevention, treatment, and diagnosis of oral cavity diseases [4]. Most dentists use bitewing radiographs to aid in the location of dental caries. They rely on information from these radiographs together with their patients' medical history. Locating of dental caries is a challenging task and sometimes even the experienced dentists miss the carious lesions when they are just presented with bitewing radiographs [5]. Traditionally, detection of dental caries relied on visual-tactile methods [6]. Sensitivity of visual-tactile methods is limited and especially done on posterior proximal teeth surfaces. Radiographic methods tend to have high sensitivity but require ionizing radiation [7].

Surveys have been carried out on various segmentation and feature extraction methods [8] that are used in preprocessing. A novel possibilistic exponential fuzzy C-means clustering algorithm proposed in [9] is used for segmenting medical images.

Analysis of dental radiographs requires some processing of the images so as to obtain useful information. The most invaluable image processing procedure or step is referred to as image segmentation. The representation of dental images is done through the segmentation of various regions of interest from the larger image so as to locate objects. Segmentation of images is therefore partitioning of an image into several segments to be used to identify objects and their edges. Image segmentation can be categorized according to similarity and discontinuity properties. Discontinuity-based methods are referred to as boundary-based methods, while similarity-based methods are referred to as region-based methods [10].

Image segmentation is the process of dividing an image into groups of similar characteristics and features. Mathematically, segmentation of an image *R* is a finite set of regions *R*1 … *R*_*s*_, *R*=∪_*i*_=1 and *R*_*i*_*R*_*i*_∩*R*_*ji*_ ≠ *j*. Research work in [11, 12] categorizes segmentation methods according to various characteristics, namely, region, entropy, shape, threshold, and pixels' correlation, among others. These characteristics were from thermal, X-ray images to aid analysis of specific points or regions of interest. Dental image segmentation is also classified as region-based, cluster-based, threshold-based, boundary-based, and watershed-based methods.

Recent advances in medical imaging analysis, especially the use of deep learning, have implemented connected component analysis to help identify, detect, classify, and quantify patterns in radiographs. At the center of these advances is the ability to explore hierarchical feature representations learned from data. Connected component analysis is pivotal to many image processing pipelines [13]. It is handled by dividing an image into foreground and background pixel objects. Then, for further processing, foreground pixels are connected to each other and extracted, while background pixels are connected together to form edges boundaries on images. Connected component analysis is used after the image has been preprocessed, and thresholding has taken place.

This paper has identified several major limitations that hinder better performances of segmentation techniques with regard to dental images. First limitation is the limited amount of dental images available for training deep learning systems. Another issue is that most dental images used are characterized with low contrast, false or fuzzy edge borders, and noise. In addition, dental images are mostly multisized, multiresolution, and multiscaled in nature. Lastly, most existing segmentation techniques require expensive computational power resources which then limit their practicability.

This proposed method is built to sort the issues or limitations aforementioned. Due to the limitation in dental images, the available 120 images have been augmented to give 11,114 images in the dataset. The augmented dataset images are then preprocessed via the Gaussian blur to remove noise. Thereafter, the erosion and dilation morphology operations are used to accentuate image pixels on the image. Lastly, segmentation is done by thresholding the pixel components connected and identified to extract the ROI of teeth. The method was trained on 10 090 training set images and tested on 1024 testing set images. An experimental analysis was done and the performance compared to state-of-the-art methods. The proposed method outperformed all of the methods in accuracy evaluation metrics.  Figure 1 shows a flow diagram of the proposed method.

## 2. Related Works

Most of the deep learning networks methods have achieved great success in segmentation of medical images. Segmentation of medical images is one of the crucial tasks in computer vision. Various researchers have proposed and developed various techniques based on deep learning networks for dental images. Some of them have been reviewed in this paper, namely, thresholding, deep convolution neural networks, and connected component analysis.

A method of identifying dead unrecognizable people is proposed in [14] using panoramic dental images. A survey of diagnosis of dental image diseases using soft computing techniques is proposed in [15]. A deep recent literature is provided in [16] covering efforts on semantic and instance segmentation. A survey of the use of the U-Net architecture is provided in [17] which is widely used in biomedical image segmentation to address the automation of identification and detection of target regions.

Soft computing techniques proposed in [18] are used to improve performance of watermarking algorithms and applications of the same. Soft computing techniques also have been adopted for segmenting images and synergistically provide malleable information competent enough to manipulate real-life circumstances. Methodologies provided in [19] are used to feat lenience for roughness, ambiguity, imprecise acumen, and partial veracity for the sake of attaining compliance and economical results.

There is also the use of the Otsu thresholding and connected component analysis proposed in [20] for the segmentation of periapical dental images to aid automated forensic identification. Connected component analysis is used to extract the region of interest (ROI) of the segmented teeth. Estimation of tooth axis in some of the existing methods requires segmenting the tooth volume from computed tornograph (CT) images; then, estimation is done from that segmented tooth volume. Poor segmentation leads to poor axis estimation [21]; thus, the estimation of molar teeth axis from two projection images is proposed rather than the segmented volume.

Connected component analysis can also be done on a set of gray levels of an image. A maximally stable extremal region (MSER) algorithm is proposed to handle this analysis. Maximal intensity regions appear to grow and merge at different intensity thresholds, while stability is achieved via finding extremal regions which are virtually unchanged over a range of threshold selection, and thus, regional intensity variation aids cyst boundary extraction in dental radiographs [22]. CNNs have been used to study consistent intensity patterns of organs at risks (OAR) from training CT images and even segment them in test CT images.

Training CNNs on CT images helps extract positive intensity patches that belong to OAR of interest and negative intensity patches that belong to surrounding structures. The patches were passed through CNN layers and image features; namely, edges, corners, and end points were captured and combined into more complex high-order features that describe the OAR efficiently. The trained network was applied to classify voxels in a ROI in the test images to obtain a corresponding OAR as a segmented image result [23].

Segmentation is a challenging task in the analysis of dental images. One of the most invaluable and yet largely unsolved issues of the level set method (LSM) is its initial contour generation. A new level set segmentation method in [24] proposes initial contour generation via morphological image information and intelligent level set segmentation through motion filtering and backpropagation of the neural network.

Early detection of dental cavity is invaluable and thus lifesaving. Ahmed et al. [25] present a caries detection method that applies *K*-means clustering and threshold method for segmentation of CT images. This is in order to construct a 3D view of the carious lesion which is an integral part of the diagnosis of dental caries. CT images have been extensively used in dental imaging diagnostics, and therefore, it is possible to use 3D data from the CT images to reconstruct 2D panoramic dental radiographs that provide a longitudinal view of the jaw bone, avoiding additional exposure to X-rays. An automatic method, introduced in [26], is used for reconstructing 2D panoramic dental images based on 3D CT images, using Bezier curves and optimization techniques, and obtained very smooth panoramic images with good contrast.

Teeth segmentation is a critical task for effective caries detection as most carious lesions usually occur around tooth boundaries, and dental images are often subject to low contrast, noise, and uneven illumination. An effective way is introduced in [27] to segment individual teeth in periapical radiographs. The method performs image enhancement via adaptive power law transformation, local singularity using Holder exponent, tooth recognition via Otsu thresholding, connected component analysis, and, lastly, tooth delineation via snake boundary tracking and morphological operations.

The accuracy of the segmentation process determines the success or failure of the final analysis process. In order to diagnose problems with wisdom teeth, Amer and Aqel [28] propose an automatic method that prepares panoramic images for segmentation, and then, a segmentation algorithm is implemented followed by a postprocessing stage, as shown by Figure 2. The preprocessing step includes contrast enhancement, Otsu thresholding, morphology operations, and connected component labeling. A segmentation algorithm was used to extract the ROI, while histogram equalization was used in the postprocessing of panoramic images.

Teeth segmentation is important in highly automated postmortem identification. Automating the process of postmortem identification using dental images has received increased attention from researchers. A mathematical morphology is offered in [29] to bitewing teeth segmentation so as to aid postmortem identification of individuals. They also propose grayscale contrast transformation and removing noise via filters for image enhancement. Next, thresholding is used to isolate teeth from the background and then group the thresholded image using connected component labeling of both background and foreground pixels to get the ROI. Finally, the connected components were refined and analyzed based on their geometric properties, and then, unqualified objects were eliminated.

An automatic approach in [30] is introduced to detect dental arches on panoramic images. They use local entropy thresholding to binarize CT images because teeth have high intensities than their surrounding areas on images. They then use connected component labeling to partially remove metal artifacts and morphological dilation to close gaps between teeth so that the mandible region is one connected piece. Finally, the thinning result gives a rough dental arch shape, and this result is exploited by a curve fitting method to get a mathematically represented dental arch.

The proposed technique uses the connected component analysis to aid teeth segmentation on dental images. Connected analysis or labeling is the process of grouping object elements of a digital image by assigning the same label to adjacent elements. This facilitates further image analysis tasks: regions can be counted and can be individually manipulated and their properties can be measured. Object labeling is important not only when dealing with large-sized images to single out and count individual regions but also when counting the number of objects in small neighborhoods. This is quite invaluable especially when designing topology preserving removal operations for thinning transformations. In 2D images, the 4-way and 8-way connected components in the special case of a 3 ^*∗*^ 3 neighborhood can be counted. The proposed technique used the 8-way connected component analysis for segmentation of dental images and is discussed in Section 3.

## 3. The Proposed Method

The proposed method proposes preprocessing and segmentation of the dental images, as shown by Figure 1, and handled by the following steps.

### 3.1. Dataset Preparation: Augmentation

With the insufficient number of dental images for research, it is impossible to derive intelligent decisions by neural networks. Deep learning networks need huge amounts of data for training and testing purposes to achieve good evaluation performance. Image augmentation is highly prescribed and involves artificially creating training images through different ways of processing or a combination of multiple processing ways on the images present. One hundred and twenty images were subjected to data augmentation techniques, namely, image shifts via the width shift range and height shift range and rotation arguments to give 11,114 images after augmentation. The data augmentation process, as discussed in [31], can be described through the following steps:

*(1) Flips.* Horizontal and vertical flips for each image in the training set. Horizontal flips are commonly used in natural images, and vertical flips are used to capture in-variance to vertical reflection in medical images.

*(2) Scaling*. We scale each one in either the *x* or *y* direction; specifically, we apply an affine transformation, *A*=(*sx*00*sy*).

*(3) Rotations*. The following affine transformation is obtained:

(1) $$\begin{array}{c} A=\left(\cos\;\theta \;\sin\;\theta -\sin\;\theta \;\cos\;\theta \right), \end{array}$$

where *θ* is between 10 and 175° and is applied.

### 3.2. Image Enhancement

Dataset preparation is first done through data augmentation; then, image enhancement is handled by improving contrast, brightness adjustment, and scaling so as to compensate the nonuniformity caused by image illumination. This is done through filtering and morphology operations. Filtering is done through the use of Gaussian blur filters to remove noise and is shown by Figure 3.

After image filtering, morphology operations that include erosion and dilation were used to diminish foreground features while accentuating background features, as shown in Figure 4.

### 3.3. Thresholding

Morphology operations in the image enhancement process was to separate teeth from the background. It is followed by image thresholding; this is used to obtain the general outline of individual teeth in the X-ray and is shown by Figure 5.

### 3.4. Connected Component Analysis

The 8-way clustering method was introduced to combine components of the same properties and neighborhood. This was after image preprocessing, image enhancement, morphology operations, and thresholding. With this method, image pixels were grouped into connected darker and brighter binary mask regions. Darker regions were combined and connected together to form the background, while brighter pixels were combined to form the foreground binary mask. This component connected analysis was used to extract the ROI shown by Figure 6.

The detection of these darker or brighter regions was influenced by the (LoG) Laplacian of Gaussian approach, which is a convolution kernel of the form

(2) $$\begin{array}{c} LoG=\frac{x^{2}+y^{2}-2\sigma^{2}}{\sigma^{4}}e^{-x^{2}=y^{2}/2\sigma^{2}}, \end{array}$$

where *σ* is the width of the kernel. The masking procedure increases segmentation accuracy.  Figure 7 shows segmentation results after the use of connected component analysis to extract the ROI on dental images.

## 4. Experiments and Results

The method was evaluated on an augmented dataset of 11,114 dental images. The dataset was split into two, the train set of 10 090 images and the test set of 1024 images. The method was trained on 10 090 train images and tested on 1024 test images. The success rate of the segmentation methods covered in this paper is from separating individual teeth from different jaw regions on an image. The success rate is measured on to how it clearly shows tooth edge boundaries and individual teeth on images throughout the whole dataset.

Teeth separation is correctly considered if the separation did not cause division of the teeth. Teeth, which were already partial as a result of being at the edge of the radiograph, are considered correctly separated if no further partiality was caused. Teeth that were not correctly segmented were either as a result of poor image contrast, where enhancement techniques could not salvage a distinction between teeth and nonteeth structures. It should be noted that the proposed segmentation method after optimization exhibited better results than compared existing implementations.  Table 1 provides a comparison of the proposed method to other implementations of connected component analysis. Results obtained from the proposed segmentation method indicate a noticeable improvement on existing models.  Figure 7 shows some image examples of the segmentation results.

Figure 8 shows training and validation accuracy graphs of the proposed threshold connected analysis segmentation method on our augmented dataset.

## 5. Conclusion and Future Work

Deep learning methods have been used for medical imaging and are now invaluable to the segmentation and detection of dental caries on dental imaging. In segmentation, regions of interest are segmented from the larger image to locate objects of similar characteristics and features. Segmentation is also the partitioning of an image into several segments from the larger image so as to locate objects and their edges. Dental image segmentation can be categorized based on similarity, namely, region-based methods, and discontinuities, namely, boundary-based methods. Several works by different authors have been reviewed to expound more on the various segmentation methods and their use.

Soft computing approaches such as fuzzy logic, artificial neural network, and genetic algorithm have been emphasized and used for image segmentation. Contribution in [32] presents state-of-the-art elaboration of almost all dimensions associated with image segmentation. They encapsulate various aspects such as emerging topics, methods, evaluation parameters, problems associated with different types of images, databases, segmentation applications, and other resources that can be advantageous to researchers in developing new methods for segmentation.

The proposed paper here has discussed the proposed threshold connected component (TCC) segmentation method used. This segmentation method used preprocessing methods that include augmentation, and image enhancement methods and thresholding were discussed and implemented to make sure accurate segmentation is achieved. Thresholding was used to obtain the general outline of teeth, and then, connected component analysis by the 8-way clustering method was used. This clustering method was used to group pixels as either dark or bright pixel masks to allow separation of teeth from the background of the whole image.

Dental image datasets are hard to find publicly; thus, there is a need for data augmentation. Evaluating performance of these deep learning methods takes longer periods due to large volumes of data and thus longer training and testing time. Several evaluation protocols for performance evaluation have been introduced to reduce the time taken for training and testing networks. Therefore, it is important to use established protocols to evaluate performance of models, networks, and methods ability to meet expectations or goals through various measurements.

There are major observations from earlier research work in the segmentation and detection of dental caries which help in making justifiable conclusions. Some of those observations that we deem very important include

- It was observed that existing work mostly employed a preprocessing step on the dental images to prepare the images for the next steps that follow
- It was also observed that the image processing method used for segmentation of dental caries had a ripple effect on the performance of the deep learning system used
- It was also observed that the performance of deep learning methods was dependent on the size of the dataset and image variability
- Data augmentation plays a big role in boosting the performance of deep learning methods especially those on not-too large datasets
- It was also observed that dental images' segmentation work use panoramic radiographs and Otsu thresholding for most connected component analysis

Therefore, it can be concluded that the proposed method provides a new approach to solve teeth segmentation problems. The method offers a robust way for providing sufficient data for deep learning in datasets through data augmentation. It also aids both individual teeth separation and edge boundary detection which makes it easier for both supervised and unsupervised learning models to correctly process teeth in the dataset. The success rate of the proposed method on the given supervised model provides a potential avenue for future work using unsupervised models thus leading to even better results.

Image analysis has been used by the proposed caries detection model in this thesis to determine presence of dental caries in dental radiographs. The final results depend heavily on the quality of the image by the time it reaches the diagnostic method. Weight regularization methods at the segmentation stage could improve the final result, and future work will look at how to implement such optimizations. The dataset that was used was relatively noise free; thus, minimal preprocessing needed to be implemented for noise removal. The dataset had few images for processing, and there was need to add more images through various processing methods, which will aid deep learning by the model. There are a series of encouraging future perspectives of study that may see improvement in dental segmentation and detection of dental caries. Among them are

- Data availability and reliability: deep learning networks require large amount of data to be able to achieve meaningful and effective performance results. Due to the nature of dental images, there is need for hybrid datasets to aid good performance of the networks. There is need of public available datasets for dental images to make deep learning possible.
- Data standardization: many methods discussed in this research are handling image preprocessing via manual methods such as cropping regions of interest on an image. These methods contribute to loss of some key details from the images. Some networks end up dividing a whole image into subregions and this ends up slowing down the learning process that occurs one subregion after the other. Other methods such as downsampling lead to deletion of important image details, and this is due to limitations in computational power. Deep learning approaches have seen an increase in learning of whole images rather than the manual manipulation of images via preprocessing, so as to get more general and accurate results.
- Weight regularization methods: deep learning methods and networks can also be improved by the introduction of weight regularization to improve their performance. The regularization of weights involves optimization of model hyperparameters such as the learning rate and the dropout rate. Basically, weight regularization methods are introduced into networks for parameter optimization.
- Hybrid approaches: deep learning methods can be further improved by combining several models or techniques to form hybrid ones that will eventually improve the overall evaluation performance. The combination can be at any stage of the model, for instance, combining two or more preprocessing techniques to come up with a single step to enhance image quality. The combination can also be handled by joining various attributes of different models to form one hybrid model that will enhance the training, extraction, detection, and classification of objects.

In addition to these optimizations, future work will look at expanding the proposed system's ability to diagnose different images, since it was used for only bitewing radiographs from the same dataset. The scope will be expanded to test a variety of different radiographic types and also bitewing radiographs from different datasets.

## Figures and Tables

**Figure 1:** Flow diagram of the proposed segmentation method.

**Figure 2:** Stages of the segmentation method with expected results from each stage [28].

**Figure 3:** Original images and images after filtering by Gaussian blur filters.

**Figure 4:** Images after erosion and dilation morphology operations.

**Figure 5:** Images after thresholding.

**Figure 6:** Masked image from the 8-way component connected clustering method.

**Figure 7:** Segmentation results of the proposed method.

**Figure 8:** Training and validation accuracy graph curves for threshold connected component analysis segmentation method, respectively.

**Table 1:** Overall comparison of segmentation methods.

Methods	Types of images	Accuracy (%)
Fuzzy C-means clustering algorithm [9]	Breast tumours' images	97.4
Local singularity analysis [27]	Periapical images	89.59
Bezier function optimization [26]	Panoramic images	91.0
Intelligent level set [24]	Periapical images	90.0
Neck segmentation using CNNs [23]	CT images	89.5
**Proposed segmentation method**	**Bitewing images**	**93.0**

The statement in bold highlights the contribution made in this paper. It is meant to distinguish the current work from related works in the literature.

## Data Availability

The data used to support the findings of the study can be obtained from the corresponding author upon request.

## Additional Points

Deep learning networks require large amount of data to be able to achieve meaningful and effective performance results. Due to the nature of dental images, there is need for hybrid datasets to aid good performance of the networks. There is need of public available datasets for dental images to make deep learning possible.

## References

[1] Kassebaum N. J., Bernabé E., Dahiya M., Bhandari B., Murray C. J. L., Marcenes W. (2015). Global burden of untreated caries. *Journal of Dental Research*.

[2] Casalegno F., Newton T., Daher R. (2019). Caries detection with near-infrared transillumination using deep learning. *Journal of Dental Research*.

[3] Schwendicke F., Dörfer C. E., Schlattmann P., Page L. F., Thomson W. M., Paris S. (2015). Socioeconomic inequality and caries. *Journal of Dental Research*.

[4] Srivastava M. M., Kumar P., Pradhan L., Varadarajan S. (2017). Detection of tooth caries in bitewing radiographs using deep learning. http://arxiv.org/abs/1711.07312.

[5] Valizadeh S., Goodini M., Ehsani S., Mohseni H., Azimi F., Bakhshandeh H. (2015). Designing of a computer software for detection of approximal caries in posterior teeth. *Iranian Journal of Radiology: A Quarterly Journal Published by the Iranian Radiological Society*.

[6] Nokhbatolfoghahaie H., Alikhasi M., Chiniforush N., Khoei F., Safavi N., Yaghoub Zadeh B. (2013). Evaluation of accuracy of DIAGNOdent in diagnosis of primary and secondary caries in comparison to conventional methods. *Journal of Lasers in Medical Sciences*.

[7] Vural U., Gökalp S. (2017). Diagnostic methods for dental caries used by private dental practitioners in Ankara. *Nigerian Journal of Clinical Practice*.

[8] Chowdhary C. L., Acharjya D. P. (2020). Segmentation and feature extraction in medical imaging: a systematic review. *Procedia Computer Science*.

[9] Chowdhary C. L., Acharjya D. P. (2017). Clustering algorithm in possibilistic exponential fuzzy C-mean segmenting medical images. *Journal of Biomimetics, Biomaterials and Biomedical Engineering*.

[10] Subramanyam R. B., Prasad K. P., Anuradha B. (2014). Different image segmentation techniques for dental image extraction. *International Journal of Engineering Research in Africa*.

[11] Sezgin M., Sankur B. (2004). Survey over image thresholding techniques and quantitative performance evaluation. *Journal of Electronic Imaging*.

[12] Silva G., Oliveira L., Pithon M. (2018). Automatic segmenting teeth in X-ray images: trends, a novel data set, benchmarking and future perspectives. *Expert Systems with Applications*.

[13] Wagner T., Lipinski H. G. (2013). IJBlob: an ImageJ library for connected component analysis and shape analysis. *Journal of Open Research Software*.

[14] Muneeswaran V., Nagaraj P., Godwin S., Vasundhara M., Kalyan G. Codification of dental codes for the cogent recognition of an individual.

[15] Rani M. P., Chopra S., Chopra J. (2021). A survey of diagnosis of dental image diseases using soft computing techniques. * International Journal for Research in Applied Science & Engineering Technology*.

[16] Minaee S., Boykov Y. Y., Porikli F., Plaza A. J., Kehtarnavaz N., Terzopoulos D. (2021). Image segmentation using deep learning: a survey. *IEEE Transactions on Pattern Analysis and Machine Intelligence*.

[17] Punn N. S., Agarwal S. (2021). Modality specific U-Net variants for biomedical image segmentation: a survey. http://arxiv.org/abs/2107.04537.

[18] Singh O. P., Singh A., Srivastava G., Kumar N. (2020). Image watermarking using soft computing techniques: a comprehensive survey. *Multimedia Tools and Applications*.

[19] Chouhan S. S., Kaul A., Singh U. P. (2019). Image segmentation using computational intelligence techniques: review. *Archives of Computational Methods in Engineering*.

[20] Chandran V., Nizar G. S., Simon P. Segmentation of dental radiograph images.

[21] Zhang D., Gan Y., Xia Z. Molar axis estimation from computed tomography images.

[22] Devi R. K., Banumathi A., Sangavi G., Dawood M. S. A novel region based thresholding for dental cyst extraction in digital dental X-ray images.

[23] Ibragimov B., Xing L. (2017). Segmentation of organs-at-risks in head and neck CT images using convolutional neural networks. *Medical Physics*.

[24] Rad A. E., Rahim M. S. M., Kolivand H., Norouzi A. (2018). Automatic computer-aided caries detection from dental x-ray images using intelligent level set. *Multimedia Tools and Applications*.

[25] Ahmed S., Saifuddin K. M., Ahmed A. S., Hossain A. A., Iqbal M. T. Identification and volume estimation of dental caries using CT image.

[26] Amorim P. H. J., Moraes T. F., Silva J. V. L., Pedrini H., Ruben R. B. (2020). Reconstruction of panoramic dental images through bézier function optimization. *Frontiers in Bioengineering and Biotechnology*.

[27] Lin P. L., Huang P. Y., Huang P. W., Hsu H. C., Chen C. C. (2014). Teeth segmentation of dental periapical radiographs based on local singularity analysis. *Computer Methods and Programs in Biomedicine*.

[28] Amer Y. Y., Aqel M. J. (2015). An efficient segmentation algorithm for panoramic dental images. *Procedia Computer Science*.

[29] Said E. H., Nassar D. E. M., Fahmy G., Ammar H. H. (2006). Teeth segmentation in digitized dental X-ray films using mathematical morphology. *IEEE Transactions on Information Forensics and Security*.

[30] Chanwimaluang T., Sotthivirat S., Sinthupinyo W. Automated dental arch detection using computed tomography images.

[31] Aggarwal s. L. P. (2019). Data augmentation in dermatology image recognition using machine learning. *Skin Research and Technology*.

[32] Chouhan S. S., Kaul A., Singh U. P. (2018). Soft computing approaches for image segmentation: a survey. *Multimedia Tools and Applications*.

